The article "Small Diameter Blood Vessels Bioengineered From Human Adipose-derived Stem Cells" was retracted in 2022. Reasons: duplicated images; unreliable results or conclusions; concerns about the data; concerns about the images.

# Small Diameter Blood Vessels Bioengineered From Human Adipose-derived Stem Cells

**DOI:** 10.1038/srep35422

**Published:** 2016-10-14

**Authors:** Renpeng Zhou, Lei Zhu, Shibo Fu, Yunliang Qian, Danru Wang, Chen Wang

**Affiliations:** 1 Department of Plastic and Reconstructive Surgery, Shanghai 9th People’s Hospital, Shanghai Jiao Tong University School of Medicine, 639 Zhi Zao Ju Road, Shanghai, 200011 P.R. China; 2 Department of Plastic & Cosmetic Surgery & Burn, The Third Affiliated Hospital of Sun Yat-sen University, 600 Tian He Road, Guangzhou, 510000, P.R. China

## Abstract

Bioengineering of small-diameter blood vessels offers a promising approach to reduce the morbidity associated with coronary artery and peripheral vascular disease. The aim of this study was to construct a two-layered small-diameter blood vessel using smooth muscle cells (SMCs) and endothelial cells (ECs) differentiated from human adipose-derived stem cells (hASCs). The outer layer was constructed with biodegradable polycaprolactone (PCL)-gelatin mesh seeded with SMCs, and this complex was then rolled around a silicone tube under pulsatile stimulation. After incubation for 6 to 8 weeks, the PCL-gelatin degraded and the luminal supporting silicone tube was removed. The smooth muscle layer was subsequently lined with ECs differentiated from hASCs after stimulation with VEGF and BMP4 in combination hypoxia. The phenotype of differentiated SMCs and ECs, and the cytotoxicity of the scaffold and biomechanical assessment were analyzed. Our results demonstrated that the two-layered bioengineered vessels exhibited biomechanical properties similar to normal human saphenous veins (HSV). Therefore, hASCs provide SMCs and ECs for bioengineering of small-diameter blood vessels.

Coronary artery and peripheral vascular disease cause death and disability worldwide. Currently, autologous or synthetic grafts are used in interventional cardiology. Autologous vessels are still the optimal approach for reconstruction of small-diameter vessels. However, the use of autologous bypass vessel graft increases the risk of secondary site injury. In the absence of adequate donor vessels, widely used synthetic grafts, such as polyethylene terephthalate (PET)^1^ and expanded polytetrafluoroethylene (ePTFE)^2^ are suitable replacements for medium (internal diameter of 6 to 10 mm, and large (diameter larger than 10 mm) vessels. Unfortunately, they do not meet the requirement for small-diameter vessels as they are prone to coagulation or thrombosis^3^ due to poor biocompatibility. Under these conditions, composite scaffolds^4^,^5^,^6^ containing biodegradable polymers blended with natural polymers provide a promising alternative. Polycaprolactone (PCL)^7^,^3^ and poly l-lactic acid (PLLA)^4^ exhibit relatively slow degradation and provide excellent mechanical properties for cell proliferation and secretion of new extracellular matrix. The synthetic materials also exhibit poor hydrophilicity and lack of cell affinity. Conversely, natural polymers, including collagen^6^ and its partial hydrolytic product (gelatin)^8^,^9^ contain several binding sites for cell adhesion and are hydrophilic. However, they display poor mechanical strength. The mixture of biodegradable synthetics with natural polymers, for example, the composite scaffold of PCL and gelatin^5^. is an effective strategy to design small-diameter vessels.

Currently, electrospinning or co-electrospinning^10^,^11^ is a promising technique for the fabrication of micro- or nano-scale fibrous scaffolds for bioengineering of vessels. This approach provides the nanofiber scaffold containing a high-surface area with high porosity for cell adhesion. However, co-electrospinning of synthetic and natural materials to develop a scaffold for bioengineered vessels remains a major challenge as the composite triggers the proliferation of cultured cells and formation of new tissue.

Several attempts have been made to utilize mature cells or different types of stem cells for blood vessel engineering. Approaches include human aortic smooth muscle cells (HASMCs)^12^, or human adipose-derived stem cells (hASCs)^13^. or coculture of vascular smooth muscle cells (SMCs) with vascular endothelial cell (ECs)^14^,^15^, or HASMCs with human umbilical vein endothelial cells (HUVECs)^16^. However, current cell types exhibit reduced expansion and unfavorable mechanical properties. A feasible and easily harvested cell source is needed.

Recently, hASCs have demonstrated the potential for differentiation into multiple cell lineages, including osteocytes, chondrocytes, smooth muscle cells and endothelial cells^7^,^8^,^9^,^10^,^11^,^12^,^13^,^14^,^15^,^16^,^17^,^18^,^19^,^20^. In addition, hASCs are easier to obtain and exhibit lower donor-site morbidity. We have demonstrated the differentiation of hASCs into SMC after induction with TGF-β1 and BMP4^21^.The newly differentiated SMCs maintain vessel architecture. Vessels bioengineered with SMCs exhibit approximately 60% of the mechanical properties of normal human saphenous veins (HSV). We, therefore, hypothesized that ECs derived from hASCs facilitate engineering of the inner layer of small-diameter vessels and serve as the main barrier to thrombosis. To fabricate a tissue engineered small-diameter vessel by culturing SMCs and ECs derived from hASCs on a degradable PCL-gelatin scaffold, we seeded SMCs on the PCL-gelatin mesh under pulsatile conditions, and seeded the ECs on the luminal surface of the smooth muscle layer to form the inner luminal lining (Fig. 1). We compared markers and biomechanical properties of the resulting two-layered bioengineered vessels under different conditions.

## Results

### Differentiation of hASCs into SMCs

The phase-contrast images of hASCs cultured in basic medium (Fig. 2A-a) and growth medium (Fig. 2A-b) showed a fine, elongated, fibroblast-like morphology. When treated with basal medium supplemented with 5 ng/mL TGF-β1 and 2.5 ng/mL BMP4 for 1 week (Fig. 2A-c), hASCs exhibited a spindle-like morphology and grew in an undulating pattern similar to the primary isolated human umbilical arterial smooth muscle cells (HUASMCs)(Fig. 2A-d). Phalloidin staining also revealed a similar fiber pattern in hASCs induced with TGF-β1 and BMP4 (Fig. 2A-c,A-d). Immunofluorescent staining of α-SMA, SM22α, calponin and SM-MHC was used to further identify the differentiation of hASCs into SMCs. In contrast to hASCs and cells cultured in basic medium (BM), only simultaneous exposure to TGF-β1 and BMP4 induced the expression of α-SMA, SM22α, calponin and SM-MHC (Fig. 2B). The differentiated hASCs (SMCs) at passage 1 showed a similar phenotype, and stained positive for α-SMA, calponin, SM22α and SM-MHC (Fig. 2C,D).

### Whole-cell patch-clamp recording

Typical currents were induced with different chemicals. Notably, the current amplitude of KCl, Ach, ET-2, ET-1 and PGF2α-induced hyperpolarization was similar in the differentiated and the hUASMCs groups. It varied significantly from that of the hASCs group (Fig. 2E and Table 1). These results confirmed that SMCs differentiating from hASCs exhibited characteristics similar to those of hUASMCs.

### Differentiation of hASCs into ECs

The hASCs generated from fresh human lipoaspirates presented endothelial-like morphology when stimulated with VEGF and BMP4 under hypoxic conditions (Fig. 3A). We further investigated the differentiation of hASCs into ECs, using immunofluorescent staining for CD31, CD144 and von Willebrand factor (vWF). Concomitant stimulation by VEGF and BMP4 under hypoxic conditions resulted in the expression of CD31, CD144 and vWF (Fig. 3B). Under normoxia, stimulation by VEGF and BMP4 did not induce uptake of low density lipoprotein from human plasma, acetylated Dil complex (DiI-Ac-LDL). However, when pharmacological stimulation was combined with hypoxia the cells absorbed DiI-Ac-LDL (Fig. 3C). Light microscopy showed a network of hUVECs similar to the differentiation of hASCs exposed to hypoxia. The hASCs grown in normoxic conditions proliferated randomly, without network formation (Fig. 3D). The nitric oxide levels in the supernatants of differentiated hASCs (ECs) after 14 days of incubation under hypoxia were also higher than in normoxia (Fig. 3E), and were comparable to levels produced by hUVECs.

### Characterization of electrospun PCL-gelatin scaffolds

The fibers were uniform in size (Fig. 4A), and SEM images showed uniform morphology of the scaffolds. The average fiber diameter was 372 ± 24 nm, with a porosity was 70.3 ± 4.3% (Fig. 4B). After culturing on fibrous scaffolds for 7 days, SMCs morphology was examined by SEM (Fig. 4C). SMCs covered the fibrous scaffolds and hybridized with the fibrous network. Cytotoxicity induced by the scaffolds was assessed by LDH leakage into the culture medium. No differences in cytotoxicity were observed between dish, membraniform and tubiform scaffolds of PCL-gelatin mesh (Fig. 4D) in cells during the 10 days of culture (Fig. 4E).

### Morphology of bioengineered vessels

The bioengineered vessels were similar to normal vessels, in that the luminal diameter was approximately 4 mm (Fig. 5A,B). H&E and Masson Trichrome staining showed that the bioengineered vessels were composed of muscle fibers in the outer layer and endothelial-like cells in the inner layer (Fig. 5C,D). Immunochemical staining showed that the outer layer was positive for α-SMA, and the inner layer was positive for CD31 (Fig. 5E, left and middle). SEM examination revealed the presence of ECs prolifeating over the lumen (Fig. 5E, right).

### Biomechanical properties

The prostaglandin I_2_ (PGI_2_) content in the pulsatile group was 219 ± 16 pg/ml, nearly 76% of the normal HSV (287 ± 16 pg/ml) and nearly 3.9 times that of the static group (56.8 ± 8.6 pg/ml) (Fig. 6A). The nitric oxide secretion in the pulsatile group was significantly higher than in the static group, approximately 81.8% that of the normal HSV (Fig. 6B, pulsatile group: 1.17 ± 0.04 μmol, normal HSV1.43 ± 0.07 μmol). The pulsatile group also contained hydroxyproline content equivalent to that of the normal vein (HSV), and significantly higher than in the static group (Fig. 6C).

The bioengineered vessel under pulsatile conditions (6.00 ± 0.78 × 10^5^ Pa) showed higher ultimate strength compared with the static group (3.07 ± 0.49 × 10^5^ Pa) (Fig. 7A). The bioengineered vessel displayed higher ultimate strain than normal HSV (Fig. 7B). No difference in elastic modulus, suture retention strength or burst pressure was found between vessels engineered under pulsatile conditions and normal HSV. The elastic modulus of the engineered vessel under pulsatile conditions (12.7 ± 1.19 MPa) was 2.76 times that of the static group (4.60 ± 0.75 MPa) (Fig. 7C). The suture retention strength of engineered vessel under pulsatile conditions was also significantly higher than in the static group (Fig. 7D, pulsatile group: 1.62 ± 0.10 N, static group: 0.58 ± 0.10 N). The engineered vessels in the pulsatile group (1.72 ± 0.14 MPa) exhibited burst pressure 3.91 times higher than that of the static group (0.44 ± 0.06 MPa), indicating superior tensile property (Fig. 7E).

## Discussion

Smooth muscle cells and endothelial cells are the main components of vasculature. We previously demonstrated that hASCs serve as a source of SMCs in blood vessel engineering^21^. Induction of hASCs with TGF-β1 and BMP-4 *in vitro* restored SMC phenotype, including expression of α-SMA, calponin and SM-MHC. After culturing the differentiated hASCs (SMCs) and PGA complexes in a bioreactor with pulsatile stimulation for 8 weeks, and assessing the ultimate strength, elastic modulus and suture retention, the bioengineered complex showed about 55% to 65% of the mechanical properties observed in normal HSV^21^. However, the absence of endothelium in previously bioengineered vessels may result in anticoagulation deficiencies. In addition, the artificial non-woven PGA scaffold represents an unorganized distribution of individual fibers.

Proliferation of endothelial cells (ECs) over the lumen of the vessel plays a potential role in the synthesis of elastin and prevention of occlusion. Synthetic vascular grafts have thrombogenic potential due to the absence of vascular endothelial cells, especially in small-diameter vessels (<6 mm)^22^. Bioengineering provides another approach to prevent earlier graft occlusion of small-diameter vessels. Human vascular smooth muscle cells^23^ or smooth muscle cells and endothelial cells isolated from the medial layer of bovine aorta^24^ are a potential source of autologous vascular cells. However, these cells exhibit insufficient proliferation, age easily and display limited ability to prevent platelet aggregation. Another promising cell source is adult mesenchymal stem cells^25^. The hASCs derived from mesoderm differentiate into multiple lineages^17^,^18^,^19^,^20^. Cao *et al.*^26^ demonstrated that hASCs showed morphology and function similar to that of endothelial cells when cultured in media containing VEGF and bFGF. According to Valdimarsdottir *et al.*^27^, the BMP pathway is potently activated in the endothelium. BMP receptor activation induces phosphorylation of specific Smad proteins and promotes EC migration and tube formation. Bekhite *et al.*^28^ demonstrated that exposure of hASCs to hypoxia in combination with leptin stimulated vascular EC differentiation. To improve structural and mechanical properties, we developed EC layers differentiated from hASCs. When stimulated by VEGF and BMP4 under hypoxia, hASCs differentiate into ECs, which are positive for CD31, CD144 and vWF. The nitric oxide production by the differentiated ECs is approximately 50% that of the hUVECs. Nitric oxide plays a potential role in thromboresistance by inhibiting platelet adhesion^29^,^30^. Compared with our previous study, the bioengineered vessels derived from the SMCs and ECs layers were analyzed histologically. Masson Trichrome staining revealed a rich, dense and organized collagen. The collagen content in the pulsatile group, based on hydroxyproline levels, was also similar to that of normal HSV. The characteristics of extracellular matrix in the two layers contributed greatly to the mechanical properties of bioengineered vessels with biomechanical strength, elastic modulus and other features similar to that of normal HSV.

Iwasaki *et al.*^31^ developed bioengineered vessels using three types of vascular cells: ECs, SMCs and fibroblasts, with equivalent strength and elasticity compared with normal HSV. However, these autogenous vascular endothelial cells showed limited potential for amplification. Du *et al.*^32^ developed a bioengineered vessel based on hUVECs, a chitosan/PCL nanofibrous vessel scaffold, and pig aorta SMCs to potentially enhance endothelial cell regeneration and anticoagulation. However, the application of hUVECs needs complex sorting, and the sorted cells need long-term cryopreservation. Conversely, hASCs show greater self-renewal, and the potential to differentiate into multiple cell types. Furthermore, adipose tissue has relatively low donor site morbidity. The hASCs are an abundant and accessible source of adult stem cells, with potential for self-renewal, differentiation and proliferation^33^.

In contrast to the bioengineered vessels under static condition, the prostaglandin PGI_2_ content in the pulsatile group was significantly higher, which inhibits platelet activation and prevention of platelet plug formation. The high nitric oxide content in the bioengineered vessels under pulsatile conditions also contributes to vascular homeostasis by inhibiting smooth muscle contraction in the endothelium, using nitric oxide to regulate the surrounding smooth muscle layer.

Electrospinning is a convenient technique for the preparation of ultrafine fibrous membranes as scaffolds due to structural similarities of the electrospun membranes with the natural extracellular matrix^17^. Compared with manual PGA scaffolds used in the previous study^21^, the electrospun PCL-gelatin scaffold fibers are uniform in size, for initial distribution of SMCs. As synthetic polymers, PCL and PGA exhibit effective mechanical properties and poor interaction with cells. The presence of gelatin in the scaffold showed superior hydrophilicity^34^, and favorable cell attachment. Previous studies showed that composite PCL-gelatin scaffolds containing 50% gelatin by weight lost structural integrity within two weeks in simulated body fluid^34^. H&E staining used in our study showed that bioengineered vessels under pulsatile conditions contained no visible scaffold by 10 weeks, and formed a dense outer muscle layer and a thin inner endothelial layer. Compared with previous bioengineered vessels under pulsatile conditions^21^(Wang C,2010), the bioengineered vessels in our study exhibit higher suture retention strength and burst pressure, which may be attributed to the organized two-layered structure and rich extracellular matrix. However, potential drawbacks include relatively complex procedure requiring 8 to 12 weeks for maturation. Further studies are needed to assess the biological function of bioengineered vessels during short-term and long-term implantation.

In summary, we have demonstrated that hASCs differentiate into cells with SMC phenotype when cultured in TGF-β1 and BMP-4. A smooth muscle layer was successfully constructed by SMCs seeded on biodegrable PCL-gelatin mesh wrapped on a silicone tube under pulsatile conditions. ECs differentiated from hASCs under hypoxia in the presence of VEGF and BMP4. Finally, we bioengineered the composite small-diameter vessels by seeding ECs on the luminal surface of smooth muscle layer to create an inner luminal lining. The novel approach may provide an effective therapeutic strategy for the management of coronary and peripheral vascular disease.

## Materials and Methods

### Human adipose-derived stem cell isolation and culture

Fresh human lipoaspirates were isolated from healthy patients following approval of the Research Ethics Committee of Shanghai Ninth People’s Hospital, as previously described^21^,^35^. All the experiments were performed in accordance with relevant guidelines and regulations and informed consent was obtained from all the patients. The hASCs were cultured in DMEM supplemented with 10% FBS (HyClone), 100 U/mL penicillin (Sigma Aldrich) and 100 mg/mL streptomycin (Sigma Aldrich), and cultured in 5% CO_2_ at 37 °C. When the cells reached 80% confluence, the cells were further passaged.

### Differentiation of hASCs (SMCs)

We previously investigated the status of isolated hASCs during differentiation under 5 ng/mL TGF- β1 (R&D Systems) and 2.5 ng/mL BMP4 (R&D Systems)^21^. The identity of SMCs was characterized by undulating morphology. They were evaluated by immunofluorescence for SMC markers. Fluorescent phallacidin (ThermoFisher, A12379) was used to label F-actin. FITC-conjugated anti-α-smooth muscle actin (αSMA), SM22α, calponin and smooth muscle-myosin heavy chain (SM-MHC) were used to identify differentiated hASCs (SMCs). When the cells reached confluence, they were subcultured and referred to as Passage 1 cells. Human umbilical artery smooth muscle cells (hUASMCs) served as the positive control.

### Whole-cell patch clamp recording

Whole-cell patch clamp recordings were performed in the current clamp mode on an inverted microscope. Currents were recorded and amplified using a HEKA patch clamp amplifier (HEKA, Germany), and pClamp 10 software (MolecularDevices, Sunnyvale, CA). A coverslip containing the attached cells was placed in the recording chamber (1 mL). Cells were continuously perfused with extracellular solution (in mmol/L: NaCl 140, KCl 5, MgCl_2_ 2, CaCl_2_ 2, HEPES 10, Glucose 10, pH 7.3–7.4). Whole cell recordings were conducted using electrodes with a resistance of about 3–5 MΩ when filled with internal solution (in mmol/L: KCl 140, HEPES 10, EGTA 5, MgCl_2_ 2.5, Mg-ATP 2, pH 7.3–7.4). Pharmacological stimuli were added to the bathing medium in the vicinity of the cell using a fast gravity perfusion system containing 80 mM KCl; 100 μM acetylcholine (Ach); 10 nM endothelin-2(ET-2); 10 nM endothelin-1(ET-1); and 100 μM prostaglandin F2α (PGF2α).

### Differentiation of hASCs (ECs) and characterization

Stimulation with 50 ng/mL VEGF and 100 ng/mL BMP4 under hypoxic conditions (37 °C, 5% CO_2_, and 2% O_2_), induced hASCs differentiation into ECs. The ECs manifested cobblestone appearance after immunofluorescence staining for CD31, CD144 and von Willebrand factor (vWF), and endothelial tube formation assay, as described previously^26^,^36^. Human umbilical vein endothelial cells (HUVECs) served as the positive control.

### Determination of LDL uptake and nitric oxide production by cultured ECs

LDL uptake was assessed by incubating cells with 2.5 μg/mL acetylated LDL labeled with Dil-Ac-LDL(Thermo Fisher, L3484), for 4 h at 37 °C. Cells were analyzed by fluorescence microscopy. Nitric oxide levels in the supernatants of differentiated hASCs (ECs) in the 14-day culture were measured using nitric acid reductase (Colorimetric Assay for Nitric Oxide, Neogen Corporation). The assays were performed by mixing 5–85 μL of supernatant with buffer to a total volume of 85 μL. Each solution was supplemented with 10 μL of the reconstituted nitrate reductase and 10 μL of 2 mM NADH, followed by incubation for 20 min at room temperature. After addition of 50 μL of Color Reagent #1 and 50 μL of Color Reagent #2, the absorbance of the sample was read at 540 nm, by spectrometry.

### Preparation of PCL-gelatin biodegradable scaffolds

The PCL-gelatin mesh (Shanghai Ju Rui Biomaterials) was used as a template for seeding of hASCs. Electrospinning solutions (5% w/v) were prepared by mixing PCL and gelatin in a weight ratio of 50:50. The electrospinning apparatus was equipped with a Statitron^®^ IFP™ power supply, which generated up to 50 KV (Tianjing High Voltage Power Supply Co., Tianjing, China). The steady flow rate of the solution was controlled at 0.7 mL/h. The electrospinning voltage was set at 16 kV. The electrospun scaffolds were collected on an aluminum foil, and vacuum-dried at room temperature for 24 h. The fiber diameter was measured based on 25 different fibers in the SEM images, and the total porosity was calculated according to previous methods^37^.

PCL-gelatin unwoven fibers were formatted into a 50 × 48 × 2 mm mesh. The scaffold was pre-sterilized with 75% ethanol, followed by overnight incubation with low glucose-DMEM (containing 10% FBS, penicillin–streptomycin). The medium was removed and the scaffold was allowed to air dry.

### Assessment of scaffold cytotoxicity

To assess the cytotoxicity induced by scaffolds, the activity of lactate dehydrogenase (LDH) in the medium was determined using a commercially available kit (Sigma Diagnostics). Cytotoxicity was calculated based on a formula provided by the manufacturer^38^. Cells were cultured with the scaffolds for 10 days, and cell counts were obtained using a Cellometer Auto T4 Cell Counter (Nexcelom).

### Seeding SMCs on PCL-gelatin scaffolds

Differentiated ASCs (SMCs) were collected and re-suspended in growth medium at a density of 5 × 10^7^ cells/mL. Each PCL-gelatin mesh in the tissue culture dishes was seeded with 1 mL of cell suspension. The cell/PCL-gelatin complexes were incubated for 4 h to allow for adhesion of cells to PCL-gelatin fibers, and the culture medium was added. The complexes were stored in an incubator for an additional 7 days, and transferred to a vessel bioreactor for further incubation.

### Pulsatile vascular bioreactor culture

The cell/PCL-gelatin complexes surrounded the silicone tubes with an outer diameter of 4 mm after 7 days in culture. In the dynamic system, the culture in the pulsatile bioreactor was performed as previously described^21^. The control samples were cultured in normal growth medium using the static culture system. The culture was maintained in the incubator at 37 °C, and the medium was refreshed every 3 days.

### Seeding differentiated hASCs (ECs) on smooth muscle cell polymer

After another 6–8 weeks of incubation, the PCL-gelatin degraded and the luminal supporting silicone tube was removed, followed by injection of 5 × 10^6^ differentiated ASCs (ECs), suspended in DMEM containing 25 mmol/L HEPES (Invitrogen), 10% FBS, 1% antibiotic-antimycotic, and 25 g/mL L-ascorbic acid, into the lumen. The outer area of the chamber was filled with the culture medium and cultured for another 1–2 weeks.

### Histology, scanning electron microscopy and immunochemistry

Tissue samples were fixed in 10% formalin, embedded in paraffin, and 5-μm-thick sections were obtained. Samples were stained with Hematoxylin and Eosin (H&E), or Masson trichrome. Other tissue samples were fixed for 30 min with 2.5% glutaraldehyde in phosphate buffer (pH 7.2). After fixation, the samples were dehydrated in a graded ethanol series. The air-dried samples were sputter coated with platinum palladium, and examined with a scanning electron microscope (SEM, Quanta 200; FEI). Immunochemical staining was performed by staining frozen cross-sections of samples fixed in cold acetone with mouse monoclonal anti-αSMA (1:100, Sigma Aldrich), and rabbit monoclonal anti-CD31 primary antibodies (1:100; Abcam), followed by incubation with the appropriate HRP-linked secondary antibody, and visualization with DAB.

### NO production, PGI_2_ and hydroxyproline content of the tubular scaffold

PGI_2_ content was measured by determining the concentration of its stable hydrolytic product. The assay was carried out according to the manufacturer’s instructions (PGI_2_ EIA kit, Cayman Chemical, Ann Arbor, MI, USA). The production of PGI_2_ was expressed as ng PGI_2_/mg protein.

Nitric oxide (NO) production was quantified using nitric acid reductase as described above, according to the manufacturer’s instructions (Colorimetric Assay for Nitric Oxide, Neogen Corporation). The absorbance of each sample was detected at 540 nm by spectrometry. The hydroxyproline content was determined using a hydroxyproline assay kit (Sigma, MAK008) to oxidize hydroxyproline with DMAB, and measure the product colorimetrically at 560 nm.

### Biomechanical assessment

The mechanical properties of the bioengineered vessel were examined as previously described^13^. Briefly, the bioengineered vessels and normal human HSV with an inner diameter of 4 mm were sectioned circumferentially. Circumferential tissue strips measuring 3 × 8 mm were mounted on a customized holder in their relaxed state. A constant elongation rate of 4 mm/min was used along the longitudinal axis of each sample. The ultimate strength and elastic modulus were analyzed according to the specimen strain and stress. Suture retention strength was measured by placing 5–0 polypropylene sutures in the four quadrants of the vessel wall, 1 mm from the vessel edge. A constant elongation force was loaded at a rate of 3 mm/min until the sutures pulled through the vessel edge. Burst pressure was tested using a pressure tester (CST1006, Const, China). The vessel was cannulated proximally, filled with PBS, and occluded distantly with a silk tie. The intraluminal pressure was increased (0.02 MPa/s) until the vessel ruptured. The burst pressure was recorded.

### Statistical analysis

Data were presented as means ± standard deviations. SPSS10.0 software was used for statistical analysis. A paired Student’s t-test was used to test the differences between the two groups. Significant differences (p-value < 0.05) are marked with asterisks in the figures.

## Additional Information

**How to cite this article**: Zhou, R. *et al.* Small Diameter Blood Vessels Bioengineered From Human Adipose-derived Stem Cells. *Sci. Rep.* **6**, 35422; doi: 10.1038/srep35422 (2016).

## Figures and Tables

**Figure 1:** Bioengineering of two-layered vessels: a schematic diagram. A PCL-gelatin mesh was seeded with SMCs and incubated for 7 days. The cell-PCL-gelatin complex was wrapped around a silicone tube. After incubation for 6–8 weeks, the PCL-gelatin degraded and the supporting tube was removed. The ECs suspended in the medium were injected into the lumen and incubated in the bioreactor culture for 1–2 weeks to develop an endothelial lining of the bioengineered vessel.

**Figure 2:** Effect of TGF-β1 and BMP4 on hASCs morphology. hASCs were cultured in BM (a), in growth medium alone (b), or in differentiation medium for 7 days (c). Primary hUASMCs served as a positive controls (d). Phalloidin staining shown in the inset of each image reveals a similar stress pattern in hASCs induced with TGF-β1 and BMP4 compared with that of primary HUASMCs. Scale bars: 50 mm for (**A–F**); 25 mm for insets. (**B**) Expression of SMC-specific proteins (α-SMA, SM22α, calponin and SM-MHC) under different culture or induction conditions. (**C**) The relative protein expression of the relevant markers under different culture or induction conditions was compared with the markers expressed in HUASMCs. Passage 1 refers to the passage cell from differentiation medium (*P < 0.05). (**D**) SMCs at passage 1 were positive for α-SMA, SM22α, calponin and SM-MHC. (**E**) The maximum currents induced by application of different chemicals. The current amplitude of hyperpolarization induced by pharmacological treatments was similar in SMCs and hUASMCs, and differed significantly from that of the hASCs group (*P < 0.05). Growth medium: DMEM + 10% FBS, BM: basic medium, DMEM + 1% FBS, Differentiation medium: DMEM + 1% FBS + 2.5 ng/ml BMP4 + 5 ng/ml TGF-β1. Data in (**C** and **E**) are expressed as mean ± SEM, n = 6.

**Figure 3:** Effect of VEGF and BMP4 under hypoxia on hASCs morphology. (**A**) In the presence of 50 ng/mL VEGF and 100 ng/mL BMP4 under hypoxia (37 °C, 5% CO_2_, 2% O_2_), hASCs manifested endothelial-like morphology. (**B**) Cells were stained with antibodies to CD31, vWF, and CD144 (green) and stained with propidium iodide (red). (**C**) Uptake of DiI-Ac-LDL (red) was assessed. (**D**) Phase-contrast image of cell tube formation; Calcein and AM staining shown in the inset of each image revealed similar results (green) (**E**) and nitric oxide concentrations. Data in E are expressed as mean ± SEM, n = 6 (*P < 0.05).

**Figure 4:** Assessment of PCL-gelatin mesh structure. (**A**) Macroscopic appearance of PCL-gelatin mesh. (**B**) SEM images show fibrous morphology of PCL-gelatin mesh. (**C**) SMCs were seeded on PCL-gelatin, and their morphology was assessed with SEM. (**D**) Toxicity of different scaffolds was assayed by measuring LDH leakage after 10 days in culture. The % LDH leakage was calculated from maximum cellular LDH leakage (N.S. not significant). (**E**) The effect of scaffolds on cell growth was assessed by counting the cell number after culture in membraniform or tubiform scaffolds for 10 days. Data in D represent mean ± SEM, n = 6. Data in E are expressed as mean ± SEM, n = 6.

**Figure 5:** Macroscopic appearance of the bioengineered vessel. (**A,B**) The luminal diameter was 4 mm. (**C,D**) Histology of the bioengineered vessels was examined using H&E staining (**C**) or Masson Trichrome staining (**D**). Both staining techniques revealed a two-layered structure, with an outer SMC layer and a luminal surface covered by ECs. (**E**) Expression of α-SMA (left) in the outer SMC layer, CD31 (middle) in the inner endothelial layer of the bioengineered vessels, and SEM images of the luminal surface of the bioengineered vessels (right)

**Figure 6:** Composition of bioengineered vessels *in vitro* under pulsatile and static conditions. (**A**) The average content of PGI_2_ in the pulsatile group was higher than in the static group. Normal HSV served as the positive control (*P < 0.05, N.S. not significant). (**B**) The average nitric oxide (NO) levels in the pulsatile group (n = 6) were higher than in the static group (*P < 0.05, N.S. not significant). (**C**) The average hydroxyproline content in the pulsatile group reached about 86% of normal HSV (*P < 0.05, N.S. not significant). P, S and N denote pulsatile group, static group and normal HSV, respectively. Data are represented as percentage changes compared with the control and are expressed as mean ± SEM, n = 6.

**Figure 7:** Comparison of mechanical properties of bioengineered vessels. Comparison of (**A**) ultimate strength, (**B**) ultimate strain (**C**) elastic modulus, (**D**) suture retention strength and (**E**) burst pressure in the pulsatile and static groups, with normal HSV serving as the positive control. P, S and N denote pulsatile, static and normal HSV groups, respectively. Data represent percentage changes compared with the normal HSV and are expressed as mean ± SEM, n = 6. (*P < 0.05, N.S. not significant).

**Table 1:** Maximal currents of cells induced by different chemicals.

Chemicals	Maximal currents (n = 25)		
	hUASMCs	Passage 1	hASCs
KCl (80 mM)	0.85 ± 0.200	0.75 ± 0.150	0.14 ± 0.020
Ach (100 μM)	0.80 ± 0.120	0.65 ± 0.130	0.10 ± 0.030
ET-2 (10 nM)	0.65 ± 0.100	0.50 ± 0.080	0.08 ± 0.001
ET-1 (10 nM)	0.62 ± 0.200	0.48 ± 0.110	0.07 ± 0.001
PGF2α (100 μM)	0.56 ± 0.110	0.45 ± 0.100	0.02 ± 0.002

Data represent mean ± SEM, n = 25.

## References

[b1] MaZ., KotakiM., YongT., HeW. & RamakrishnaS. Surface engineering of electrospun polyethylene terephthalate (PET) nanofibers towards development of a new material for blood vessel engineering. Biomaterials 26, 2527–2536 (200).1558525510.1016/j.biomaterials.2004.07.026

[b2] LordM. S., YuW., ChengB., SimmonsA., Poole-WarrenL. & WhitelockJ. M. The modulation of platelet and endothelial cell adhesion to vascular graft materials by perlecan. Biomaterials 30, 4898–4906 (2009).1954058710.1016/j.biomaterials.2009.05.063

[b3] PektokE. *et al.* Degradation and healing characteristics of small-diameter poly(epsilon-caprolactone) vascular grafts in the rat systemic arterial circulation. Circulation 118, 2563–2570 (2008).1902946410.1161/CIRCULATIONAHA.108.795732

[b4] ShalumonK. T., DeepthiS., AnupamaM. S., NairS. V., JayakumarR. & ChennazhiK. P. Fabrication of poly (L-lactic acid)/gelatin composite tubular scaffolds for vascular tissue engineering. Int J Biol Macromol 72, 1048–1055 (2015).2531641810.1016/j.ijbiomac.2014.09.058

[b5] FuW. *et al.* Electrospun gelatin/PCL and collagen/PLCL scaffolds for vascular tissue engineering. Int J Nanomedicine 13, 2335–2344 (2014).10.2147/IJN.S61375PMC402655424872696

[b6] Heydarkhan-HagvallS. *et al.* Three-dimensional electrospun ECM-based hybrid scaffolds for cardiovascular tissue engineering. Biomaterials 29, 2907–2914 (2008).1840301210.1016/j.biomaterials.2008.03.034PMC2397445

[b7] AllenR. A. *et al.* Nerve regeneration and elastin formation within poly(glycerol sebacate)-based synthetic arterial grafts one-year post-implantation in a rat model. Biomaterials 35, 165–173 (2014).2411945710.1016/j.biomaterials.2013.09.081PMC3882022

[b8] LamprouD., ZhdanP., LabeedF. & LekakouC. G elatine and gelatine/elastin nanocomposites for vascular grafts: processing and characterization. J Biomater Appl. 26, 209–226 (2011).10.1177/088532821036442920566658

[b9] PereiraI. H. *et al.* Differentiation of human adipose-derived stem cells seeded on mineralized electrospun co-axial poly(epsilon-caprolactone) (PCL)/gelatin nanofibers. J Mater Sci Mater Med. 25, 1137–1148 (2014).2437884810.1007/s10856-013-5133-9

[b10] BakerB. M., HandorfA. M., IonescuL. C., LiW. & J. MauckR. L. New directions in nanofibrous scaffolds for soft tissue engineering and regeneration. Expert Rev Med Devices 6, 515–532 (2009).1975112410.1586/erd.09.39PMC2828681

[b11] ZhengR. *et al.* The influence of Gelatin/PCL ratio and 3-D construct shape of electrospun membranes on cartilage regeneration. Biomaterials 35, 152–164 (2014).2413526910.1016/j.biomaterials.2013.09.082

[b12] VatankhahE., PrabhakaranM. P., SemnaniD., RazaviS., MorshedM. & RamakrishnaS. Electrospun tecophilic/gelatin nanofibers with potential for small diameter blood vessel tissue engineering. Biopolymers 101, 1165–1180 (2014).2504200010.1002/bip.22524

[b13] WangC., GuoF., ZhouH., ZhangY., XiaoZ. & CuiL. Proteomic profiling of tissue-engineered blood vessel walls constructed by adipose-derived stem cells. Tissue Eng Part A. 19, 415–425 (2013).2296335010.1089/ten.tea.2011.0532PMC3542882

[b14] LiH., LiuY., LuJ., WeiJ. & LiX. Micropatterned coculture of vascular endothelial and smooth muscle cells on layered electrospun fibrous mats toward blood vessel engineering. J Biomed Mater Res A. 103, 1949–1960 (2015).2520430610.1002/jbm.a.35332

[b15] ZhangH. *et al.* Dual-delivery of VEGF and PDGF by double-layered electrospun membranes for blood vessel regeneration. Biomaterials 34, 2202–2212 (2013).2329046810.1016/j.biomaterials.2012.12.005

[b16] ShinoharaS. *et al.* Fabrication of *in vitro* three-dimensional multilayered blood vessel model using human endothelial and smooth muscle cells and high-strength PEG hydrogel. J Biosci Bioeng 116, 231–234 (2013).2352338210.1016/j.jbiosc.2013.02.013

[b17] MajumdarM. K., BanksV., PelusoD. P. & MorrisE. A. Isolation, characterization, and chondrogenic potential of human bone marrow-derived multipotential stromal cells. J Cell Physiol. 185, 98–106 (2000).1094252310.1002/1097-4652(200010)185:1<98::AID-JCP9>3.0.CO;2-1

[b18] HalvorsenY. D. *et al.* Extracellular matrix mineralization and osteoblast gene expression by human adipose tissue-derived stromal cells. Tissue Eng. 7, 729–741 (2001).1174973010.1089/107632701753337681

[b19] WangC. *et al.* Differentiation of adipose-derived stem cells into contractile smooth muscle cells induced by transforming growth factor-beta1 and bone morphogenetic protein-4. Tissue Eng Part A. 16, 1201–1213 (2010).1989520510.1089/ten.TEA.2009.0303

[b20] GaafarT. M., Abdel RahmanH. A., AttiaW., HamzaH. S., BrockmeierK. & El HawaryR. E. Comparative characteristics of endothelial-like cells derived from human adipose mesenchymal stem cells and umbilical cord blood-derived endothelial cells. Clin Exp Med. 14, 177–184 (2014).2364987510.1007/s10238-013-0238-5

[b21] WangC. *et al.* A small diameter elastic blood vessel wall prepared under pulsatile conditions from polyglycolic acid mesh and smooth muscle cells differentiated from adipose-derived stem cells. Biomaterials 31, 621–630 (2010).1981954510.1016/j.biomaterials.2009.09.086

[b22] WiseS. G., ByromM. J., WaterhouseA., BannonP. G., WeissA. S. & NgM. K. A multilayered synthetic human elastin/polycaprolactone hybrid vascular graft with tailored mechanical properties. Acta Biomater 7, 295–303 (2011).2065607910.1016/j.actbio.2010.07.022

[b23] DahlS. L. *et al.* Readily available tissue-engineered vascular grafts. Sci Transl Med. 3, 68ra9 (2011).10.1126/scitranslmed.300142621289273

[b24] NiklasonL. E. *et al.* Functional arteries grown *in vitro*. Science 284, 489–493 (1999).1020505710.1126/science.284.5413.489

[b25] KhanW. S. & HardinghamT. E. Mesenchymal stem cells, sources of cells and differentiation potential. J Stem Cells 7, 75–85 (2012).23550346

[b26] CaoY., SunZ., LiaoL., MengY., HanQ. & ZhaoR. C. Human adipose tissue-derived stem cells differentiate into endothelial cells *in vitro* and improve postnatal neovascularization *in vivo*. Biochem Biophys Res Commun 332, 370–379 (2005).1589670610.1016/j.bbrc.2005.04.135

[b27] ValdimarsdottirG. *et al.* Stimulation of Id1 expression by bone morphogenetic protein is sufficient and necessary for bone morphogenetic protein-induced activation of endothelial cells. Circulation 106, 263–270 (2002).10.1161/01.cir.0000033830.36431.4612390958

[b28] BekhiteM. M. *et al.* Hypoxia, leptin, and vascular endothelial growth factor stimulate vascular endothelial cell differentiation of human adipose tissue-derived stem cells. Stem Cells Dev. 23, 333–351 (2014).2413462210.1089/scd.2013.0268

[b29] MajorT. C. *et al.*The mediation of platelet quiescence by NO-releasing polymers via cGMP-induced serine 239 phosphorylation of vasodilator-stimulated phosphoprotein. Biomaterials 34, 8086–8096 (2013).2390651410.1016/j.biomaterials.2013.07.041PMC3771351

[b30] IrwinC., RobertsW. & NaseemK. M. Nitric oxide inhibits platelet adhesion to collagen through cGMP-dependent and independent mechanisms: the potential role for S-nitrosylation. Platelets 20, 478–486 (2009).1985268610.3109/09537100903159375

[b31] IwasakiK. *et al.* Bioengineered three-layered robust and elastic artery using hemodynamically-equivalent pulsatile bioreactor. Circulation 118, S52–S57 (2008).1882476910.1161/CIRCULATIONAHA.107.757369

[b32] DuF. *et al.* Gradient nanofibrous chitosan/poly varepsilon-caprolactone scaffolds as extracellular microenvironments for vascular tissue engineering. Biomaterials 33, 762–770 (2012).2205628510.1016/j.biomaterials.2011.10.037

[b33] GimbleJ. M., KatzA. J. & BunnellB. A. Adipose-derived stem cells for regenerative medicine. Circ Res. 100, 1249–1260 (2007).1749523210.1161/01.RES.0000265074.83288.09PMC5679280

[b34] BinulalN. S., NatarajanA., MenonD., BhaskaranV. K., MonyU. & NairS. V. PCL-gelatin composite nanofibers electrospun using diluted acetic acid-ethyl acetate solvent system for stem cell-based bone tissue engineering. J Biomater Sci Polym Ed. 25, 325–340 (2014).2427410210.1080/09205063.2013.859872

[b35] CuiL., YinS., LiuW., LiN., ZhangW. & CaoY. Expanded adipose-derived stem cells suppress mixed lymphocyte reaction by secretion of prostaglandin E2. Tissue Eng. 13, 1185–1195 (2007).1751870410.1089/ten.2006.0315

[b36] ArnaoutovaI. & KleinmanH. K. *In vitro* angiogenesis: endothelial cell tube formation on gelled basement membrane extract. Nat Protoc. 5, 628–635 (2010).2022456310.1038/nprot.2010.6

[b37] ChenH. *et al.* Electrospun chitosan-graft-poly (ɛ-caprolactone)/poly (ɛ-caprolactone) nanofibrous scaffolds for retinal tissue engineering. Int J Nanomedicine 6, 453–461 (2011).2149943410.2147/IJN.S17057PMC3075910

[b38] FotakisG. & TimbrellJ. A. *In vitro* cytotoxicity assays: comparison of LDH, neutral red, MTT and protein assay in hepatoma cell lines following exposure to cadmium chloride.Toxicol Lett. 160, 171–177 (2006).1611184210.1016/j.toxlet.2005.07.001

